The article "Wearable Devices and Intelligent Application in Women's Postpartum Repair for Smart Healthcare" was retracted in 2023. Reasons: signs of a paper mill; suspected computer-generated content; unreliable results or conclusions; concerns about the data.

# Wearable Devices and Intelligent Application in Women's Postpartum Repair for Smart Healthcare

**DOI:** 10.1155/2022/4454926

**Published:** 2022-01-07

**Authors:** Jing Wang, Danfeng Wang

**Affiliations:** ^1^Operation Room of Gynaecology OutPatient, the First People's Hospital of Wenling, Taizhou 317500, China; ^2^Recovery Room of Anesthesiology Department, the First People's Hospital of Wenling, Taizhou 317500, China

## Abstract

Wearable devices are more and more widely used in the field of smart healthcare. The purpose of this study was to explore the effect of contraceptive counseling and education on contraceptive behavior of women after induced abortion. The investigators will explain the situation of this topic to the respondents and select the respondents in strict accordance with the framework requirements of sampling design. All the data are from the induced abortion women in the first-, second-, and third-level hospitals, which reduces the selection bias of the respondents. It is found that the proportion of induced abortion among college students is the highest, reaching 66.03%. This study is helpful to reduce the incidence of unwanted pregnancy, induced abortion, and repeated abortion and improve the reproductive health of women.

## 1. Introduction

Wearable devices are more and more widely used in the field of smart healthcare. It is the most natural physiological need. In many primitive languages, sex and eating are expressed in the same word. Visibility, like eating, is the most basic activity of human beings. Sexual behavior is the basic link of ethnic continuity, but also has the function of enjoyment, and is an important form of human life fun. As far as abortion is concerned, there are four trends in China: high rate of abortion, rising rate of unmarried pregnancy, low age of abortion, and high rate of repeated abortion.

Before the “two child” policy, China's family planning policy was very tough. In recent years, with the rapid development of economy, the accelerated pace of life, the increase of floating population, and the change of sexual concept, after the “two child” policy, the contraceptive methods of women of childbearing age also changed, which led to the increase in unplanned pregnancy rate; the better living conditions made people put eugenics in an important position. In addition, the weak awareness of self-protection and the lack of understanding of the harm of abortion are also one of the important reasons for the rate of induced abortion.

Abortion accounts for 10% of Ghana's maternal mortality rate, and it is a serious health problem. Helena et al. believe that in order to accelerate progress towards the Millennium Development Goal 5, abortions must be drastically reduced. The barriers to contraceptive use are due to concerns about side effects, inconveniences, socioeconomic factors, bad social norms, and poor service provision. Although this research has not met the high demand for family planning, the research process is too complicated [1]. Tohma et al. explored the predictive value of transvaginal ultrasound symptom assessment in the diagnosis of residual products of pregnancy (RPOC) after artificial negative pressure voluntary termination of pregnancy. Although this study can diagnose the sensitivity of RPOC on the 7th day, the study lacks comparative data [2]. Rasti et al. believe that ToRCH infection is related to poor obstetric prognosis. However, there is little information on the impact of ToRCH co-infection on pregnancy outcomes. Therefore, they tested *Toxoplasma gondii* in 81 pregnant women with abortion (case group) and 98 pregnant women with normal delivery (control group). Although this research can show that in the single infection model, only the CMV-IgM seropositivity rate is significantly higher than that of the control group, the pattern recognition in the co-infection model is not very clear [3]. Perri et al. believe that the debate on the relationship between modern contraception and abortion in population policy has long existed. They studied Nepal's legalization of abortion regulations in 2004 and subsequent expansion of abortion services, an unusual and quickly implemented policy that meets these requirements, using four waves of rich personal level data representing the age of conception of Nepalese women. Although their findings have important implications for public policy and foreign aid, they did not propose effective strategies to reduce expensive and potentially unsafe abortions [4].

The article "Wearable Devices and Intelligent Application in Women's Postpartum Repair for Smart Healthcare" was retracted in 2023. Reasons: signs of a paper mill; suspected computer-generated content; unreliable results or conclusions; concerns about the data.

The objective is to understand the stakeholders' acceptance of “promoting PAFP service in all levels and types of hospitals and family planning institutions”; to collect the “opportunities and challenges of implementing PAFP service after the establishment of the Health and Family Planning Commission” mentioned by stakeholders; to collect the possible obstacles and ways of PAFP service policy transformation proposed by stakeholders. The investigators will explain the situation of this topic to the respondents and select the respondents in strict accordance with the framework requirements of sampling design. All the data are from the induced abortion women in the first-, second-, and third-level hospitals, which reduces the selection bias of the respondents.

## 2. Women's Contraception

### 2.1. Abortion

The advantage of surgical abortion is that it can solve the problem in the shortest time and with the fastest efficiency. However, with clinical application, it has been found to have more complications and adverse reactions. Compared with medical abortion, its recent complications are easier when the menopause time is longer; causes bleeding; and due to uterine deformity or excessive flexion, it is easy to cause perforation [5, 6]. Its advantage is to avoid the above adverse reactions and complications, the patient's psychological burden is less, and the pain degree is relatively low [7]. The safe and effective termination of unintended pregnancy is essential [8, 9]. People not only demand to relieve the patient but also put the safety and effectiveness of the treatment method in a higher position in the process of disease diagnosis and treatment [10].

### 2.2. Medical Abortion

It analyzes the current situation of unmarried adolescents' abortion from different aspects such as their own reasons, family reasons, and social reasons [11, 12]. From the physical, psychological, and social harm caused by artificial abortion to adolescents, it makes a specific analysis and proposes intervention measures from China's national conditions, family, society, community, and hospitals [13].

Assume that an existing data stream signs the message of a certain node [14, 15]. Then,

(1) Rsourse=⊕i=0k−1Signaturei⊕Timestramp,Q=Str To IntSub Str End32HmodMQ,

in which, *Q* is a random number. Then, each node is voted with the probability of PI [16]:

(2) $$\begin{array}{c} P1=\frac{K}{M\;d}. \end{array}$$

Then, assuming that each node gets Y signatures with probability *P*2, we can get [17, 18]

(3) $$\begin{array}{c} P2=C_{MW}^{Y}*\left(\frac{K}{M\;d}\right)*{\left(1-\frac{K}{M\;d}\right)}^{M\;d-Y}. \end{array}$$

Assuming that the probability of being successfully selected as a production node is *P*3, we get [19]

(4) $$\begin{array}{c} P3=\sum_{i=Mw/2}^{Mw}\frac{Mw!}{\left(i!\left(Mw-i\right)!\right)}*{\left(\frac{K}{M\;d}\right)}^{i}*{\left(1-\frac{K}{M\;d}\right)}^{Mw-i}. \end{array}$$

Then, let *P*4 be the probability that a candidate node is successfully selected as a production node [20, 21], namely,

(5) $$\begin{array}{c} P4=\frac{Mq}{M\;d},\\ f\left(X_{i}\left(k\right)\right)=\frac{X_{i}\left(k\right)}{A\left(k\right)},\\ X_{i}=\left(X_{1i},X_{2i},\ldots ,X_{ji}\right),\;i=1,2,\ldots ,n. \end{array}$$

When *P*3=*P*4, K can be calculated [22].

### 2.3. Sexuality

Throughout history, society's attitude towards sex is like a continuum from strict confinement to extreme openness. One end is the attitude of sexual prohibition and strict control of sexual behavior, while the other end is sexual liberation, sexual indulgence, and advocacy. The attitude of complete sexual freedom is dominated. These two extreme attitudes are detrimental to human physical and mental health and the healthy development of the society [23, 24]. With the rapid development of the country's economy in recent years and the rapid development of IT technology, the concept of young people has become more and more influenced by Western culture. Sexual openness and even sex, indulgent films, books, and Internet information can be seen everywhere. When the open environment of sex collides with the lack of sex education, the mystification of sex by traditional concepts arouses young people's curiosity about sex, and the lack of access to education makes them choose more self-exploration or nonprofessional channels [25, 26]. Ignorance and misunderstanding of sex and reproduction and bad sexual hygiene habits are the consequences of the disconnect between education and the environment. Many unmarried women become pregnant because of the lack of sexual knowledge in a sexually open environment [27, 28].

The article "Wearable Devices and Intelligent Application in Women's Postpartum Repair for Smart Healthcare" was retracted in 2023. Reasons: signs of a paper mill; suspected computer-generated content; unreliable results or conclusions; concerns about the data.

## 3. Experiment on the Influence of Women's Contraceptive Behavior

### 3.1. Research Objects

Inclusion criteria: during the survey period, from May 2018 to October 2020, women who were diagnosed with pregnancy at the study site and requested termination of pregnancy; understand the current situation of PAFP policy and service development in the area where some stakeholders (health policy makers, medical and health institution managers, health service providers, and health policy researchers) are located; understand stakeholders' opinions on “in all levels and types of hospitals and the acceptance of the promotion of PAFP services by family planning agencies; collection of “opportunities and challenges in implementing PAFP services after the establishment of the Health and Family Planning Commission” mentioned by stakeholders; collection of possible obstacles and approaches to the transformation of PAFP service policies mentioned by stakeholders.

### 3.2. Research Design

The items in the questionnaire were determined by a procedural decision-making method. The decision-making group composed of patients undergoing induced abortion, obstetricians and gynecologists, health education experts, and statistical experts.

Sex-related behaviors: age and reason for first sex, number of sexual partners, frequency of sexual behavior, frequency and type of contraception, reasons for not using contraception every time, etc.

### 3.3. Sampling Design

This survey was a stratified sampling, and the survey subjects were from first-, second-, and third-level hospitals. The number of independent variables included in the survey table was 80, taking 10–20 times. Combined with pre-investigation and analysis of stratification factors such as the number of people in tertiary hospitals, it was finally determined that about 2,000 cases were sampled in tertiary hospitals, 1,000 cases in second-level hospitals, and 282 cases in first-level hospitals.

The article "Wearable Devices and Intelligent Application in Women's Postpartum Repair for Smart Healthcare" was retracted in 2023. Reasons: signs of a paper mill; suspected computer-generated content; unreliable results or conclusions; concerns about the data.

### 3.4. Investigation Implementation

#### 3.4.1. Interview Design

The survey project was verified by ethics experts and passed. The method of current situation research was adopted, and the self-made questionnaire improved after preliminary investigation was used to obtain the data of the research object.

The interviews were conducted on a one-to-one basis. In order to improve the quality of interviews, recordings were made with the consent of the interviewees. The interviewer recorded relevant information during the interview and immediately proofread and improved the content of the interview with the interviewee after the interview. Another interviewer independently recorded the content of the interview based on the audio recording. Two interviewers checked and compared and recorded the results and made a summary of the interview together. The investigation site was set up in the waiting room and rest room for patients before and after induced abortion. There were no family members and other unrelated persons or onlookers during the investigation.

The thematic framework analysis method was used to process interview data. The interview data were entered into the computer and manually marked. The theme framework was determined by repeatedly reading the interview outline and interview materials. The information was classified, analyzed, and summarized by subject, to sort out the barriers to the transformation of PAFP (post-abortion family planning) service policy, related information, and other content from the perspective of interviewees.

#### 3.4.2. Questionnaire Design

1. Based on literature research, interview results, and expert opinions, the main ways of PAFP service policy transformation were preliminarily determined, and questionnaires were made;
2. Experts in the field of post-abortion health care were invited to conduct a technical review of the questionnaire;
3. The completed electronic questionnaire was sent in the form of WeChat, QQ group, and e-mail;
4. The person who filled in the form was invited to conduct “completely unfeasible,” “not feasible,” “generally feasible,” “relatively feasible,” “completely feasible,” and “unclear” for each possible path in each aspect one by one; determination of dimensions was done;
5. The questionnaire was automatically retrieved by the system after filling in. A total of 552 questionnaires were collected and 552 were valid questionnaires (electronic questionnaires that did not meet the valid conditions could not be submitted), and the questionnaire efficiency was 100%. The software background was used to collect questionnaire data, and statistical software was used to enter the data. The basic information of survey subjects and their choices of different transformation methods was sorted through statistical description, whether there are differences and differences in the choices of different types of survey subjects were examined, and a basis for proposing specific transformation methods and their priority in implementation was provided.

The article "Wearable Devices and Intelligent Application in Women's Postpartum Repair for Smart Healthcare" was retracted in 2023. Reasons: signs of a paper mill; suspected computer-generated content; unreliable results or conclusions; concerns about the data.

### 3.5. Quality Control

Data source: the investigator explained the situation of the subject to the survey subjects and strictly abided by the sampling design framework requirements to select the survey subjects. All the data are from the abortion women in the first-, second-, and third-level hospitals, reducing the number of subjects. The questionnaire was adjusted according to the results of the pre-survey. The questionnaire was designed with a closed-ended selection sentence structure. The questions were simple and clear and easy to answer to reduce nonresponse bias; the investigators have been uniformly trained to respond to the questions. Consistent understanding reduces the interobserver variation; the inquiry tone strives to be unified and reduces the intraobserver variation. Data input method: all data adopt EpiData3.1 double recording method, after using SPSS21.0 statistical software, exploratory exploration, analyze and logically check, find unreasonable data, analyze the reasons, and ensure the correctness of the data for analysis.

## 4. Women's Contraceptive Behavior

### 4.1. Basic Situation of the Research Object

The degree of anxiety of unmarried women undergoing abortion (48.79 + 7.81) and the degree of anxiety of married women undergoing abortion (40.70 + 9.23) were tested with independent samples: *t* = −5.668, *p* < 0.01; similarly, depression score in the unmarried group (50.91 + 8.84) and the depression score of the married group (41.54 + 10.54) were tested by the independent sample *t* test, *t* = 5.687, *p* < 0.01. It can be seen that there are extremely significant differences between the unmarried group and the married group in the degree of anxiety and depression of women who have also induced abortion. The rates of repeated abortions for married and unmarried women are shown in Table 1.

Correlation analysis of the three dimensions of social support for unmarried women with induced abortion and SAS score shows that subjective support, support utilization, and total social support scores are not related to anxiety levels, but objective support levels and anxiety levels are significant. Negative correlation: *r* = −0.392, *p*=0.009 < 0.01; that is, the more the objective support an individual receives, the lower the anxiety level. Similarly, the level of objective support is also significantly negatively correlated with the degree of depression: *r* − 0.369, *p*=0.015 < 0.05. The higher the degree of objective support an individual receives, the lower the level of anxiety and depression. The analysis of the causes of miscarriage is shown in Figure 1.

The article "Wearable Devices and Intelligent Application in Women's Postpartum Repair for Smart Healthcare" was retracted in 2023. Reasons: signs of a paper mill; suspected computer-generated content; unreliable results or conclusions; concerns about the data.

The five personality characteristics of unmarried women with induced abortion are correlated with the three categories and total scores of social support as bivariates. Cautiousness, extraversion, and openness are positively correlated with social objective support, and neuroticism is negative with objective social support. The three dimensions of attribution tendency of unmarried women with induced abortion are correlated with the three categories and total scores of social support as bivariates, and there is no significant correlation, indicating that the attribution method has no correlation with social support.  Table 2 shows the statistics of bleeding, menstrual recovery, abdominal pain, and fever one month after the operation. The analysis result is shown in Figure 2.

Researchers should strengthen communication with health policy makers and form research reports into easy-to-understand forms, such as short and capable policy briefs, and submit them to health policy makers. The presentation of data and policy recommendations should be emphasized in research reports, and key information should be provided. Researchers should start from the aspects that are of interest to health policy makers, connect the work of health policy transformation with specific functional departments, and propose a set of specific and feasible plans for health policy makers to adopt. 265 aborted women aged 20–44 years. In addition, the study found that college students accounted for the highest proportion, reaching 66.03%.  Table 3 shows the distribution of women's economic income and educational level of abortion. The distribution of education level is shown in Figure 3.

### 4.2. Abortion Women's Awareness of Contraceptive Knowledge

The survey found that more people obtain sexual knowledge through the Internet, accounting for 71%. Therefore, it is very important for PAFP service policy transformation to popularize PAFP services and correct misconceptions. Some people, such as unmarried people and floating population, have great demand for PAFP services, but the existing service provision for these people is insufficient; coupled with their own special needs, they need to pay special attention to PAFP service policy transformation. Therefore, early education on sexual health of young people should be promoted, and the role of parents should be emphasized in youth education. In schools, counseling and peer education can be carried out through youth health education clubs or similar institutions. In terms of propaganda and education materials, professional institutions or departments can provide core contraceptive education information, and various regions can develop educational propaganda materials suitable for different populations according to the characteristics of different populations. At the same time, attention should be paid to the publicity of contraceptive knowledge by the mass media, especially strengthening the supervision and regulation of network publicity, to ensure that the public obtains accurate and sufficient information. In addition, attention should be paid to male health education and male participation in PAFP.  Figure 4 shows the way to acquire knowledge about contraception.

The article "Wearable Devices and Intelligent Application in Women's Postpartum Repair for Smart Healthcare" was retracted in 2023. Reasons: signs of a paper mill; suspected computer-generated content; unreliable results or conclusions; concerns about the data.

## 5. Conclusion

Wearable devices are more and more widely used in the field of smart healthcare. Relieving unmarried abortion women's bad psychological problems is only one aspect of the problem of unmarried abortion. We must look at this social issue that has received much attention from a more comprehensive and macro perspective, and we must start from the origin of the problem. Only by preventing unmarried first pregnancy can we truly reduce the abortion rate and promote the development of reproductive health and social health.

Education on sexual ethics and sexual concepts should be strengthened for unmarried young people through multiple channels from schools, families, hospitals, communities, media, and relevant government departments, sexual and reproductive health information and services should be provided, safe, healthy, and responsible sexual behavior should be promoted, and scientific research should be conducted. The contraceptive guidance correctly guides teenagers to face their own behaviors and improve self-protection awareness, thereby reducing the possibility of unmarried teenagers' unintended pregnancy and fundamentally reducing the rate of miscarriage and reproductive tract diseases.

However, they are in a weak position in the material wealth and power distribution of the entire society, which restricts their autonomy. However, on the psychological and spiritual level, adolescents show the characteristics of free running, and it is even difficult to be restrained by society. Their autonomy is more sufficient than that of adults and young children. “Under such circumstances, it is recommended that basic education should be used.” “Sexual purity education” and “sex safety education” should be combined. However, it does not mean that premarital sex must be strictly prohibited. It should be based on correct sexual hygiene knowledge and consciously prevent unwanted pregnancy and prevent sexually transmitted diseases.

The article "Wearable Devices and Intelligent Application in Women's Postpartum Repair for Smart Healthcare" was retracted in 2023. Reasons: signs of a paper mill; suspected computer-generated content; unreliable results or conclusions; concerns about the data.

## Figures and Tables

**Figure 1:** Analysis of the causes of abortion.

**Figure 2:** Analysis results.

**Figure 3:** Distribution of educational level.

**Figure 4:** Approaches of cognitive acquisition of contraceptive knowledge.

**Table 1:** Repeated abortion rates among married and unmarried women.

Marital status	Number of repeated abortions	Single abortion
Married	1000 (46.79%)	1137 (53.21%)
Unmarried	441 (38.52%)	704 (61.48%)

**Table 2:** Partial statistical results of 1-month follow-up after surgery.

In a month	The total number	The number of follow-up	Bleeding time	Unrecovered menstruation
	(people)	(people)	(days)	(people)
Sep 2018	192	156 (81.25%)	4.97	1
In October 2018	247	212 (85.83%)	5.18	1
In November 2018	260	229 (88.08%)	6.02	6
In December 2018	274	227 (82.85%)	6.14	2

**Table 3:** Distribution of economic income and educational level of women with induced abortion.

Parameter	General situation	Numbers	Percentage
Average monthly income	<2000 yuan	84	31.7
	2000–5000 yuan	150	56.60
	>5000 yuan	31	11.69
Level of education	Below junior high school	16	6.04
	High school, technical school, technical school	52	19.62
	College or undergraduate	175	66.04
	Postgraduate and above	22	8.30

## Data Availability

The data used to support the findings of this study are included within the article.

## References

[1] Agyei H., Otupiri E., Larson-Reindorf R. E. (2016). Preventing repeat abortions among women in Kumasi, Ghana. *American Journal of Public Health Research*.

[2] Tohma Y. A., Dilbaz B., Evliyaoğlu Ö., Çoşkun B., Çolak E., Dilbaz S. (2016). Is ultrasonographic evaluation essential for diagnosis of retained products of conception after surgical abortion?. *Journal of Obstetrics and Gynaecology Research*.

[3] Rasti S., Ghasemi F. S., Abdoli A., Piroozmand A., Mousavi S. G. A., Fakhrie-Kashan Z. (2016). ToRCH “co-infections” are associated with increased risk of abortion in pregnant women. *Congenital Anomalies*.

[4] Perri P. F., Pelle E., Stranges M. (2016). Estimating induced abortion and foreign irregular presence using the randomized response crossed model. *Social Indicators Research*.

[5] Miller G., Valente C. (2016). Population policy: abortion and modern contraception are substitutes. *Demography*.

The article "Wearable Devices and Intelligent Application in Women's Postpartum Repair for Smart Healthcare" was retracted in 2023. Reasons: signs of a paper mill; suspected computer-generated content; unreliable results or conclusions; concerns about the data.

[6] Vu Q., Micks E., McCoy E., Prager S. (2016). Efficacy and safety of long-acting reversible contraception in women with cardiovascular conditions. *The American Journal of Cardiology*.

[7] Moniz M. H., Chang T., Davis M. M., Forman J., Landgraf J., Dalton V. K. (2016). Medicaid administrator experiences with the implementation of immediate postpartum long-acting reversible contraception. *Women’s Health Issues*.

[8] Meckstroth K. R., Darney P. D. (2000). Implantable contraception. *Obstetrics & Gynecology Clinics of North America*.

[9] Schwenkhagen A. M., Stodieck S. R. G. (2008). Which contraception for women with epilepsy?. *Seizure*.

[10] Mørch L. S., Skovlund C. W., Hannaford P. C., Iversen L., Fielding S., Lidegaard Ø. (2017). Contemporary hormonal contraception and the risk of breast cancer. *New England Journal of Medicine*.

[11] Gubrium A. C., Mann E. S., Borrero S. (2016). Realizing reproductive health equity needs more than long-acting reversible contraception (LARC). *American Journal of Public Health*.

[12] Beauchamp A. (2016). Abortion costs, separation, and non-marital childbearing. *Journal of Family and Economic Issues*.

[13] Grossman D., White K., Hopkins K., Potter J. E. (2017). Change in distance to nearest facility and abortion in Texas, 2012 to 2014. *JAMA*.

[14] Moniz M., Chang T., Heisler M., Dalton V. K. (2017). Immediate postpartum long-acting reversible contraception: the time is now. *Contraception*.

[15] Athas W. F., Adams-Cameron M., Hunt W. C., Amir-Fazli A., Key C. R. (2000). Travel distance to radiation therapy and receipt of radiotherapy following breast-conserving surgery. *Journal of the National Cancer InstituteJournal of the National Cancer Institute*.

[16] Kaur R., Gupta K. (2016). Endocrine dysfunction and recurrent spontaneous abortion: an overview. *International Journal of Applied and Basic Medical Research*.

[17] Bongaarts J. (2017). The effect of contraception on fertility: is sub-Saharan Africa different?. *Demographic Research*.

[18] Lawton B., Makowharemahihi C., Cram F., Robson B., Ngata T. (2016). Pounamu: E Hine: access to contraception for indigenous Mãori teenage mothers. *Journal of Primary Health Care*.

[19] Espey E., Ogburn T. (2011). Long-acting reversible contraceptives. *Obstetrics & Gynecology*.

[20] Wang R.-W., Dunn D. W., Sun B. F. (2014). Discriminative host sanctions in a fig-wasp mutualism. *Ecology*.

[21] Hall K. S., McDermott Sales J., Komro K. A., Santelli J. (2016). The state of sex education in the United States. *Journal of Adolescent Health*.

[22] Weatherly J. N., Plumm K. M., Derenne A. (2011). Delay discounting and social policy issues. *Psychological Record*.

The article "Wearable Devices and Intelligent Application in Women's Postpartum Repair for Smart Healthcare" was retracted in 2023. Reasons: signs of a paper mill; suspected computer-generated content; unreliable results or conclusions; concerns about the data.

[23] Vesce F., Giugliano E., Bignardi S. (2014). Vaginal lactoferrin administration before genetic amniocentesis decreases amniotic interleukin-6 levels. *Gynecologic and Obstetric Investigation*.

[24] Sun X., Qian F., He Y., Gu X., Di W. (2020). Safety and efficacy of combined oral contraceptive ethinyl estradiol/drospirenone (YAZ) in Chinese women: a single-arm, open-label, multicenter, post-authorization study. *Advances in Therapy*.

[25] Yu H., Zhao Y., Liu Z. (2021). Research on the financing income of supply chains based on an E-commerce platform. *Technological Forecasting and Social Change*.

[26] Liu Z., Lang L., Li L., Zhao Y., Shi L. (2021). Evolutionary game analysis on the recycling strategy of household medical device enterprises under government dynamic rewards and punishments. *Mathematical Biosciences and Engineering: MBE*.

[27] Cohen G. L., Aronson J., Steele C. M. (2000). When beliefs yield to evidence: reducing biased evaluation by affirming the self. *Personality and Social Psychology Bulletin*.

[28] Daaleman T. P. (2016). Primary care of adults with intellectual and developmental disabilities. *Southern Medical Journal*.

